The article "Chai-Hu-San-Shen Capsule Ameliorates Ventricular Arrhythmia Through Inhibition of the CaMKII/FKBP12.6/RyR2/Ca2+ Signaling Pathway in Rats with Myocardial Ischemia" was published in 2022. Journal: Evid Based Complement Alternat Med.

# Chai-Hu-San-Shen Capsule Ameliorates Ventricular Arrhythmia Through Inhibition of the CaMKII/FKBP12.6/RyR2/Ca^2+^ Signaling Pathway in Rats with Myocardial Ischemia

**DOI:** 10.1155/2022/2670473

**Published:** 2022-10-03

**Authors:** Longqing Chen, Rongzhen Liu, Weisong Wang, Congcong Tang, Junning Ran, Wei Huang, Shuqi Li, Jianhe Liu

**Affiliations:** ^1^Department of Cardiology, The First Hospital of Hunan University of Chinese Medicine, Changsha 410007, China; ^2^Department of Traditional of Chinese Medicine, The Fourth Hospital of Changsha, Changsha 410006, China

## Abstract

Ventricular arrhythmia is one of the main causes of sudden cardiac death, especially after myocardial ischemia. Previous studies have shown that Chai-Hu-San-Shen capsule (CHSSC) can reduce the incidence of ventricular arrhythmias following myocardial ischemia, however, the mechanisms of it are unclear. In present study, we explored the mechanism of CHSSC ameliorates ventricular arrhythmia following myocardial ischemia via inhibiting the CaMKII/FKBP12.6/RyR2/Ca^2+^ signaling pathway. *In vivo*, a myocardial ischemia rat model was established and treated with CHSSC to evaluate the therapeutic effect of CHSSC. *In vitro*, we established an ischemia model in H9C2 cells and treated with CHSSC, KN-93, or H-89. Then, intracellular Ca^2+^ content, the expression of RyR2, and the interaction between FKBP12.6 and RyR2 were detected. The results showed that CHSSC could delay the occurrence of ventricular arrhythmias and shorten the duration of ventricular arrhythmias. After myocardial ischemia, the intracellular Ca^2+^ content was increased, and CHSSC treatment mitigated this increase, down-regulated the levels of p-CaMKII, CaMKII, p-RyR2, and RyR2, and up-regulated the levels of p-RyR2 (Ser2808) and p-RyR2 (Ser2814). Co-immunoprecipitation showed an interaction between FKBP12.6 and RyR2, and CHSSC up-regulated the content of the FKBP12.6-RyR2 complex in ischemic cells. In conclusion, our study showed that CaMKII activation led to hyperphosphorylation of RyR2 (Ser2814) and RyR2 (Ser2808) during cardiomyocyte ischemia, which resulted in dissociation of the FKBP12.6-RyR2 complex, and increased intracellular Ca^2+^ content, which may contribute to the development of ventricular arrhythmias. CHSSC may reduce the incidence of ventricular arrhythmias following myocardial ischemia through inhibition of the CaMKII/RyR2/FKBP12.6/Ca^2+^ signaling pathway.

## 1. Introduction

Arrhythmia is an important factor in cardiovascular diseases. Mild arrhythmias typically result in no obvious negative impact on human health, but the occurrence of ventricular arrhythmia often leads to sudden death [1]. Acute ischemic arrhythmia is a major cause of sudden cardiac death. Although modern medicine has resulted in improvements in the treatment of arrhythmia, better treatment strategies are needed. A large body of literature supports traditional Chinese medicine (TCM) as a successful treatment strategy for arrhythmia. However, a large number of TCM prescriptions are available, and most of the mechanisms of these medicines are not clear. Therefore, it is of great theoretical value and clinical significance to identify a prescription that improves ventricular arrhythmias following myocardial ischemia, and to determine the mechanisms by which this improvement occurs.

The article "Chai-Hu-San-Shen Capsule Ameliorates Ventricular Arrhythmia Through Inhibition of the CaMKII/FKBP12.6/RyR2/Ca2+ Signaling Pathway in Rats with Myocardial Ischemia" was published in 2022. Journal: Evid Based Complement Alternat Med.

Reperfusion injury after myocardial ischemia can lead to different types of arrhythmias [2, 3], which are closely related to the abnormal autonomic activity triggered by the imbalance of intracellular Ca^2+^ [4]. Intracellular Ca^2+^ is mainly derived from the sarcoplasmic reticulum (SR) of striated muscle and the endoplasmic reticulum (ER) in other types of cells, and is regulated by Ca^2+^ release channels located on the SR/ER, including Reynolds Ryanodine receptors (RyRs, including RyR1, RyR2, and RyR3) [5]. RyR2 is mainly expressed in the myocardium, and plays a key role in the E-C coupling process of cardiomyocytes though the regulation of intracellular Ca^2+^ concentration [6]. Activation of RyR2 results in release of SR Ca^2+^ into the cytoplasm. The concentration of Ca^2+^ increases rapidly, causing myocardial contraction. Subsequently, the Ca^2+^-ATPase located on the SR is activated, which results in energy expenditure to pump Ca^2+^ back into the SR, which results in myocardial diastole [7].

Studies have shown that activation of CaMKII can be detected in the initial stage of cardiac ischemia/reperfusion [8, 9], and activation of CaMKII can result in RyR2 channel opening through phosphorylation of Ser2814 on RyR2, thereby increasing SR Ca^2+^ release, which regulates myocardial contraction [4]. In addition, FKBP12 and FKBP12.6 are also involved in modulation of RyR2 activity by binding to RyR2 protein, which contributes to Ca^2+^ homeostasis. Ryanodine receptor R2 has a higher affinity for FKBP12.6 than for FKBP12 [10]. Binding of FKBP12.6 to the RyR2 channel results in formation of a complex that can promote closure of the RyR2 channel, resulting in inhibition of release of SR Ca^2+^ [11]. Myocardial ischemia, or other disease factors, result in dissociation of the FKBP12.6 and RyR2 complex. This dissociation results in activation and opening of the RyR2 channel, leading to a rapid increase in Ca^2+^ concentration in the cytoplasm. This rapid increase can trigger abnormal potentials and cause arrhythmia [11, 12]. Dissociation of FKBP12.6 and RyR2 may result from hyperphosphorylation of RyR2 (Ser 2808) by PKA [12, 13].

The article "Chai-Hu-San-Shen Capsule Ameliorates Ventricular Arrhythmia Through Inhibition of the CaMKII/FKBP12.6/RyR2/Ca2+ Signaling Pathway in Rats with Myocardial Ischemia" was published in 2022. Journal: Evid Based Complement Alternat Med.

Our previous studies showed that Chai-Hu-San-Shen capsule (CHSSC) can be used effectively to treat coronary heart disease ventricular premature contraction, through reduced expression of CaMKII and through modulation of sarcoplasmic reticulum calcium ATPase activity [14–17]. However, the effects of CHSSC downstream of CaMKII are unclear. In this study, we established a rat model of ischemic arrhythmia to characterize the therapeutic effects of CHSSC and the influence of CHSSC on the CaMKII/FKBP12.6/RyR2/Ca^2+^ signaling pathway. We also established a H9C2 cell model of myocardial ischemia to detect changes in intracellular Ca^2+^ content, the expression of RyR2, and the interaction between FKBP12.6 and RyR2 to evaluate the effects of CHSSC on ventricular arrhythmia after myocardial ischemia through regulation of the CaMKII/FKBP12.6/RyR2/Ca^2+^ signaling pathway.

## 2. Materials and Methods

### 2.1. Preparation of CHSSC

Chai-Hu-San-Shen capsule was provided by the Pharmaceutical Preparation Room of the First Hospital of Hunan University of Chinese Medicine (lot#: 20181127). The Chinese herbs used in CHSSC are presented in Table 1. Contents of the capsule were dissolved in normal saline at a concentration of 0.43 g/mL for use.

### 2.2. Medicated Plasma of CHSSC and Nonmedicated Plasma

Ten Sprague Dawley (SD) rats were randomly divided into two groups for the preparation of medicated plasma and nonmedicated plasma. The medicated plasma group was given CHSSC at 0.43 g/dose twice per day for 3 days. The nonmedicated plasma group was given the same dose of normal saline. On the fourth day, blood was collected following treatment of CHSSC or normal saline for 0.5, 1, 2, 3, and 5 h, and then centrifuged. All the rats were fasted, but allowed water ad libitum, for 12 h before blood collection.

### 2.3. Reagents

Anti-CaMKII (#4436S) and anti-p-CaMKII (#12716S) were purchased from Cell Signaling Technology, Inc. (Massachusetts, USA). Anti-RyR2 (#ab2868) and anti-p-RyR2 (Ser2808) (#ab59225) were purchased from Abcam (Cambridge, UK). Anti-p-RyR2 (Ser2814) (#ap0624) was from ABclonal Technology Co., Ltd. (Wuhan, China). Anti-FKBP12.6 (#sc-376135) was from Santa Cruz Biotechnology (Shanghai, China). CaMKII inhibitor KN-93 (#S7423) and PKA inhibitor H-89 (#S1582) were from Selleck Biotechnology Co., Ltd. (Shanghai, China). Horseradish peroxidase goat antirabbit IgG (#ZB-2301), and HRP goat antimouse IgG (#ZB2305) were from Beijing Zhongshan Jinqiao Biotechnology Co., Ltd. (Beijing, China).

### 2.4. Animals

Forty 8-week-old SD male rats (body weight 200 ± 20 g) were purchased from Changsha Tianqin Biotechnology Co., Ltd. [certification NO.: SYXK (Xiang) 2013–0005]. All rats were sheltered in cages at a room temperature of 25°C with a 12 h light/dark cycle [certification no: SCXK (Xiang) 2015–0003]. Experimental animals were allowed access to drinking water ad libitum. All animal experiments were conducted in accordance with the National Institutes of Health (NIH) Guide for the Care and Use of Laboratory Animals No. 80–26 and ARRIVE guide, and were approved by the Ethics Committee for Experimental Animals of The First Hospital of Hunan University of Chinese Medicine.

The article "Chai-Hu-San-Shen Capsule Ameliorates Ventricular Arrhythmia Through Inhibition of the CaMKII/FKBP12.6/RyR2/Ca2+ Signaling Pathway in Rats with Myocardial Ischemia" was published in 2022. Journal: Evid Based Complement Alternat Med.

### 2.5. H9C2 Cell

H9C2 cells (#ZQ0102) were purchased from Shanghai Zhongqiaoxinzhou Biotech Co., Ltd. (Shanghai, China). After recovery, culture, and cryopreservation, the H9C2 cells were grown to about 90% confluence and continuously cultured for further experiments.

### 2.6. Animal Grouping and Modeling

After adaptive feeding for one week, rats were randomly divided into a sham operation group (Sham), a myocardial ischemia model group (Control), a CHSSC treatment group (CHSSC), and a CaMKII inhibitor KN-93 treatment group (KN-93). Each group was administered the indicated treatment for 10 consecutive days before ligation of the left anterior descending coronary artery. Ligation was performed 30 min after the final administration. The specific administration methods and doses were as follows: CHSSC: 0.86 g/d, i.g [18]; KN-93 : 5 mg/kg, i.p, once every 2 days [19]. The sham and the model group were given the same amount of normal saline by gavage, respectively.

After the final administration, the rats were anesthetized, and the whole lead II ECG was recorded using a biological signal collector. The trachea was opened and connected to a ventilator, after which the skin was cut longitudinally at the left edge of the sternum, and the tissues were separated successively to expose the heart and to separate pericardium. The left anterior descending coronary artery was ligated using a needle inserted from the lower edge of the left atrial appendage. Successful ligation was indicated by significantly elevated ST segment from lead II, a high T wave, and darkened color of the heart surface below the ligation line. After ligation for 30 min, ECG changes were observed following infusion. The anesthesia and thoracotomy for the sham operation were the same as those for the model group, ECG was recorded, but no ligation was performed. Rats were removed from the study if they exhibited abnormal ECG before ligation, coronary artery ligation failed or no reperfusion was observed, excessive bleeding, or heart beat and breath stopped for more than 30 s.

The article "Chai-Hu-San-Shen Capsule Ameliorates Ventricular Arrhythmia Through Inhibition of the CaMKII/FKBP12.6/RyR2/Ca2+ Signaling Pathway in Rats with Myocardial Ischemia" was published in 2022. Journal: Evid Based Complement Alternat Med.

### 2.7. H9C2 Cell Grouping and Modeling

A myocardial ischemia model was established in H9C2 cells using an ischemic solution. The composition of the solution was NaH_2_PO_4_ 0.028 g; NaHCO_3_ 0.1008 g; MgSO_4_ 0.0592 g; Sodium lactate 0.897 g; HEPES 1.042 g; NaCl 1.151 g; KCl 0.149 g; and CaCl_2_ 0.0399 g. These components were dissolved in 200 mL of ultra-pure water, and the pH was adjusted to 6.5 using concentrated hydrochloric acid. The solution was then filtered through microporous membranes (0.22 *μ*m). The experiment was started when the cardiomyocytes neared confluence and showed synchronous pulsation. The normal culture medium was replaced with the ischemic solution, and the cells were placed in a sealed gas container filled with 95% N2/5% CO_2_ for 3 h.

The following groups were used for the first experiment. Cells were randomly divided into the following groups: control group (Control), model group (Model), CHSSC treatment group (CHSSC), and CaMKII inhibitor KN-93 treatment group (KN-93). The control group was cultured normally without any treatment. The model group underwent simulated ischemia. Following ischemia, the medium in the CHSSC group was replaced with fresh medium and plasma containing CHSSC (10%, 200 *μ*l) was added, and the cells were incubated for 48 h. The KN-93 group received KN-93 (1 *μ*M, 0.04 *μ*l) for 1 h prior to establishment of the ischemia model. The medium was replaced following the ischemic period.

The following groups were used for the second experiment. H9C2 cells were randomly divided into control cell + H-89 group (Control + H-89), ischemia model + H-89 group (Model + H-89), ischemia model + H-89 + nonmedicated plasma group (Model + H-89 + plasma), ischemia model + H-89 + CHSSC medicated plasma group (Model + H-89 + CHSSC), and ischemia model + H-89 + KN-93 group (Model + H-89+KN-93). The treatments in each group were as follows. The Control + H-89 group received H-89 (5 *μ*M, 1 *μ*l) for 1 h, followed by replacement with a fresh medium. The Model + H-89 group received H-89 (1 *μ*M, 1 *μ*l) 1 h prior to establishment of the ischemia model for 3 h, followed by replacement with a fresh medium. The Model + H-89 + plasma group received H-89 (5 *μ*M, 1 *μ*l) for 1 h prior to establishment of the ischemia model for 3 h. The medium was then replaced, nonmedicated plasma (10%, 200 *μ*l) was added, and the cells were cultured for 48 h. The Model + H-89 + CHSSC group received H-89 (5 *μ*M, 1 *μ*l) for 1 h prior to establishment of the ischemia model for 3 h. The medium was replaced and CHSSC-medicated plasma (10%, 200 *μ*l) was added. The cells were cultured for 48 h. The Model + H-89 + KN-93 group received H-89 (1 *μ*M, 1 *μ*l) and KN-93 (1 *μ*M, 0.04 *μ*l) for 1 h prior to establishment of the ischemia model. The medium was then replaced with a fresh medium.

The article "Chai-Hu-San-Shen Capsule Ameliorates Ventricular Arrhythmia Through Inhibition of the CaMKII/FKBP12.6/RyR2/Ca2+ Signaling Pathway in Rats with Myocardial Ischemia" was published in 2022. Journal: Evid Based Complement Alternat Med.

### 2.8. Electrocardiogram Recording and Ventricular Arrhythmia Score

An RM-6280 biological signal acquisition system was used to monitor ECG, and lead II was recorded. The frequency and first occurrence time of ventricular premature beat (VPB) and the frequencies and durations of ventricular tachycardia (VT) and ventricular fibrillation (VF) were recorded in each group after ligation.

### 2.9. Determination of Optimal Medicated Plasma Concentration Using MTT Assay

Cells were washed twice with a preheated RPMI1640 medium, and a mononuclear cell suspension was prepared with RPMI1640 nutrient solution containing fetal bovine serum. The cells were seeded at 2×10^5^ cells/mL (100 *μ*l/well) in 96-well plates. The cells were then treated with 5, 10, or 20 *μ*l of CHSSC medicated plasma or nonmedicated plasma, which resulted in final concentrations of 5%, 10%, and 20%, respectively. Each concentration was evaluated in triplicate. The plates were then incubated in a 5% CO_2_ atmosphere at 37°C for 48 h. Twenty microliters (5 g/L) of MTT solution was added to each well, and the cells were incubated for 4 h. The supernatant was removed, and 200 *μ*l of DMSO was added to each well and the plates were shaken for 10 min. Using 630 nm wavelength as the reference, the absorbance (OD) value for each well was determined at 492 nm. The medicated cells which had the highest survival rate were used to determine the intervention concentration for subsequent experiments. Survival rate = mean OD value of CHSSC medicated plasma treated group/mean OD value of normal group × 100%.

### 2.10. Flow Cytometry Assay

Cells were washed twice with PBS, then centrifuged at 111 ×  *g* for 5 min. Diluted calcium ion solution (calcium ion stock solution concentration was 5 mM, and the working concentration was 5 *μ*M) was used to resuspend cell pellets. The cells were incubated in a dark environment at 37°C for 30 min, with mixing every 3–5 min. Then, the cell pellets were collected and washed twice with a serum-free medium. Within 1 h, the green fluorescence of Ca^2+^-FITC (excitation wavelength Ex = 488 nm, emission wavelength Em = 530 nm) was detected using flow cytometry through the FITC channel (FL1).

### 2.11. Western Blot

Cells were lysed on ice, then centrifuged at 16000 × *g* for 15 min at 4°C to obtain the supernatant. The protein concentration was measured using a BCA protein quantitation kit. An 8% separation gel and 4.8% loading gel were prepared, and the gels were poured following addition of TEMED. For each sample, 120 *μ*l of protein supernatant was combined with 30 *μ*l of 5× loading buffer, and the solution was mixed well and boiled for 5 min. The samples were then placed on ice until use. Electrophoresis was performed with a constant voltage of 75V for 130 min, which was the time required for bromophenol blue to reach the bottom of the gel. At 300 mA constant current, RyR2, p-RyR2 (Ser2808), and p-RyR2 (Ser2814) were transferred for 150 min and *β*-actin was transferred for 60 min onto nitrocellulose membranes. After transfer, the membrane was placed at room temperature for 60 min, then incubated at 4°C overnight. The membranes were incubated with primary antibodies [diluted with 1 × as follows: RyR2, 1 : 6000; p-RyR2 (Ser2808), 1 : 3000; p-RyR2 (Ser2814) 1 : 5000; and *β*-actin, 1 : 5000] at room temperature for 90 min. The membranes were then washed with 1 × PBST 3 times, then incubated with secondary antibodies (diluted with 1× PBST as follows: HRP goat antimouse IgG, 1 : 5000; HRP goat antirabbit IgG, 1 : 6000) at room temperature for 90 min. The membranes were then washed with 1 × PBST three times, then incubated with ECL chemiluminescence solution for 1 min for detection.

The article "Chai-Hu-San-Shen Capsule Ameliorates Ventricular Arrhythmia Through Inhibition of the CaMKII/FKBP12.6/RyR2/Ca2+ Signaling Pathway in Rats with Myocardial Ischemia" was published in 2022. Journal: Evid Based Complement Alternat Med.

### 2.12. Co-Immunoprecipitation Assay

After washing with PBS, 300 *μ*l of IP lysate was added to the cell pellets. The pellets were ultrasonicated, and then centrifugated at 16000 × *g* for 15 min at 4°C to obtain the supernatant. The supernatant was divided and antibody (A, which was prepared by taking 40 *μ*l from each of the 5 samples: normal mouse IgG 3 *μ*l; B, which was IP lysate: mouse-derivedanti-FKBP12.6 10 *μ*l; C, which was holoprotein: no antibody) was added and mixed. Then, 200 *μ*l of IP lysate was added to 20 *μ*l of protein A/G agarose beads and mixed, and then centrifuged 4 times at 1000 × *g* for 3 min to obtain precipitates. The IP lysate incubated overnight with antibody was then added to the pretreated Protein A/G agarose beads and slowly shaken at 4°C for 2 h for conjugation. After co-immunoprecipitation, the mixtures were centrifuged at 1000 × *g* for 3 min to obtain supernatants. Western blot experiments were performed according to Section 2.11.

### 2.13. Statistical Analysis

All data in this paper are expressed as the mean ± standard deviation (SD). For normally distributed data, Student's t-test was used for statistical comparison between two groups, and one-way ANOVA was used to compare differences among three or more groups. Post-hoc Fisher's least significant difference (LSD) test or Dunnett's test were used for individual group comparisons. *P* < 0.05 was considered statistically significant. Statistical analysis was performed using SPSS 25.0 software.

The article "Chai-Hu-San-Shen Capsule Ameliorates Ventricular Arrhythmia Through Inhibition of the CaMKII/FKBP12.6/RyR2/Ca2+ Signaling Pathway in Rats with Myocardial Ischemia" was published in 2022. Journal: Evid Based Complement Alternat Med.

## 3. Results

### 3.1. Effect of CHSSC on Electrocardiogram and Ventricular Arrhythmia Score in Rats with Myocardial Ischemia

As shown in Figure 1, the sham operation group did not exhibit ventricular arrhythmia (Figure 1(a)). The model group, CHSSC treatment group, and KN-93 treatment group all showed ventricular arrhythmia (Figures 1(b)–1(d)). As shown in Table 2, the rats had low VPB and VF frequency, later first occurrence time of VPB, and shorter VT duration following treatment with CHSSC or KN-93 when compared with the model group.

### 3.2. Effect of CHSSC on Protein Expression of CaMKII, p-CaMKII, RyR2, And p-RyR2 in Rats with Myocardial Ischemia

To further explore the mechanism of CHSSC against arrhythmia, western blot was used to determine the levels of CaMKII, p-CaMKII, RyR2, and p-RyR2 in the myocardial tissue of each group. As shown in Figure 2, the levels of CaMKII, p-CaMKII, RyR2, and p-RyR2 in the model group were significantly up-regulated compared with those in the sham operation group (Figures 2(b)–2(e)). Following intervention with CHSSC or the CaMKII inhibitor KN-93, the levels of CaMKII, p-CaMKII, and RyR2, were significantly lower than those in the model group, but higher than those in the sham operation group, which indicated that both CHSSC and CaMKII inhibitor KN-93 down-regulated the expression of CaMKII, p-CaMKII, RyR2, and p-RyR2 in myocardial tissue of rats with myocardial ischemia.

### 3.3. Effect of CHSSC on Intracellular Ca^2+^ Content in Ischemic H9C2 Cells

Abnormally increased calcium ion concentration in myocardial cells is an important contributor arrhythmia. We established a myocardial cell ischemia model by simulating ischemia in H9C2 myocardial cells, and used flow cytometry to detect changes in intracellular Ca^2+^ content in each group. We determined the survival rate of H9C2 cells using the MTT assay to determine the optimal CHSSC plasma concentration. As shown in Table 3, H9C2 cells in the 5% medicated plasma group had the highest survival rate, while the 20% medicated plasma group had the lowest, which suggested that 5% medicated plasma was the optimal CHSSC medicated plasma for subsequent experiments. As shown in Figure 3, compared with the control group, the fluorescence intensity in the model group was significantly increased. Compared with the model group, the CHSSC treatment group and KN-93 group both exhibited weaker fluorescence signal. This indicated that intracellular Ca^2+^ content was significantly increased following ischemia, and treatment with CHSSC or the CaMKII inhibitor KN-93 mitigated this increase.

### 3.4. Effects of CHSSC on H9C2 Cell RyR2, p-RyR2 (Ser2808), and p-RyR2 (Ser2814) in Ischemic H9C2 Cell

Hyperphosphorylation of p-RyR2 (Ser2808) and p-RyR2 (Ser2814) is an important contributor to arrhythmia induced by abnormal RyR2 function. Western blot was used to determine the expression levels of RyR2, p-RyR2 (Ser2808), and p-RyR2 (Ser2814) in each group. As shown in Figure 4, the levels of RyR2 did not differ among the groups. However, the levels of p-RyR2 (Ser2808) and p-RyR2 (Ser2814) were significantly increased in the model group compared with those in the control group. Furthermore, the levels of p-RyR2 (Ser2808) were significantly decreased, and a downward nonsignificant trend for p-RyR2 (Ser2814) was observed following treatment with CHSSC medicated plasma or KN-93. These results suggested that myocardial ischemia can induce phosphorylation at Ser2808 and Ser2814 on RyR2, and CHSSC and the CaMKII inhibitor KN-93 may regulate the opening of Ca^2+^ channels by inhibiting activation of Ser2808 on RyR2 following myocardial ischemia.

The article "Chai-Hu-San-Shen Capsule Ameliorates Ventricular Arrhythmia Through Inhibition of the CaMKII/FKBP12.6/RyR2/Ca2+ Signaling Pathway in Rats with Myocardial Ischemia" was published in 2022. Journal: Evid Based Complement Alternat Med.

### 3.5. Effect of CHSSC on the Interaction Between FKBP12.6 and RyR2 in Ischemic H9C2 Cell

The results in Section 3.4 indicated that CHSSC can inhibit up-regulation of p-RyR2 (Ser2808) and p-RyR2 (Ser2814) in H9C2 cells after ischemia. We evaluated whether CHSSC induced dissociation of the FKBP12.6-RyR2 complex as a protective mechanism against arrhythmia. Co-immunoprecipitation was used to detect the interaction between FKBP12.6 and RyR2 in each group. As shown in Figure 5, the expression level of FKBP12.6 did not differ among the groups. However, the expression of RyR2 was significantly decreased following ischemia compared with that in the control group. Furthermore, the expression of RyR2 was up-regulated following intervention with CHSSC medicated plasma or KN-93 when compared with that in the model + H-89 group and model + H-89 + nonmedicated plasma groups. These results suggested that there is an interaction between FKBP12.6 and RyR2 protein, and that dissociation of the FKBP12.6-RyR2 complex occurred in response to myocardial ischemia. Treatment with CHSSC or the CaMKII inhibitor KN-93 prevented dissociation of this complex.

## 4. Discussion

Arrhythmia is a common cardiovascular disease, and ventricular arrhythmias such as ventricular premature beat, ventricular tachycardia, and ventricular fibrillation can lead to sudden cardiac death [20–26]. Ventricular arrhythmias induced by myocardial ischemia or ischemia-reperfusion are often missed or ignored, but can be life-threatening [27]. A large number of traditional Chinese medicines have been used to treat ischemic arrhythmias with results. These include Wenxin granule [28] and Shensong Yangxin capsule [29], composed of Bupleuri Radix, Pinelliae Rhizoma Praeparatum, Salviae Miltiorrhizae Radix Et Rhizoma, Codonopsis Radix, Sophorae Flavescentis Radix, Coptidis Rhizoma, Artemisiae Annuae Herba, and Glycyrrhizae Radix Et Rhizoma. CHSSC is a Chinese traditional formula based on the traditional TCM pathogenesis of “Shaoyang disorder” with the treatment goal of “harmonize and release the Shaoyang.” Our previous studies showed that CHSSC can antagonize experimental arrhythmias induced by chloroform, calcium chloride, and aconitine in a dose-dependent manner [18]. A clinical study found that CHSSC effectively reduced the number of VPB [30]. Studies have shown that CHSSC can reduce the incidence of ventricular arrhythmias following myocardial ischemia in rats through increased expression of SERCA2a and decreasing Ca^2+^ concentration in myocardial cells [16]. In this study, our data showed that there were no ventricular arrhythmias in the sham operation group, but obvious ventricular arrhythmias occurred after myocardial ischemia. Intervention with CHSSC or the CaMKII inhibitor KN-93 significantly reduced the frequency of VPB and VT, delayed the time to the appearance of VPB, and shortened the duration of VF. These results indicated that CHSSC significantly inhibited ventricular arrhythmia in rats with myocardial ischemia, which highlighted the importance of determining the mechanisms of action of this medication.

The article "Chai-Hu-San-Shen Capsule Ameliorates Ventricular Arrhythmia Through Inhibition of the CaMKII/FKBP12.6/RyR2/Ca2+ Signaling Pathway in Rats with Myocardial Ischemia" was published in 2022. Journal: Evid Based Complement Alternat Med.

Since Ringer first observed that cardiac contraction requires Ca^2+^ in 1988, the role of Ca^2+^ as a signaling ion in the heart has been studied extensively, and Ca^2+^ imbalance has been shown to play a key role in the pathogenesis of cardiovascular diseases, including arrhythmias [31–33]. Studies have shown that CHSSC can delay the time to onset of arrhythmias and shorten the duration of arrhythmias by reducing the concentration of Ca^2+^ in cardiomyocytes of rats with myocardial ischemia [17]. We established a myocardial ischemia model by simulating ischemia in H9C2 cells using a simulated ischemic solution, and found that CHSSC significantly mitigated ischemia-induced increases Ca^2+^ content. This effect may be related to the involvement of CHSSC in regulation of CaMKII and RyR2 activation. The SR is the main location of intracellular calcium storage in muscle cells [34], and Ca^2+^ release from the SR is mediated by RyR2, a specific Ca^2+^ release channel [35–37]. Increased Ca^2+^ leakage from the SR through the RyR2 channel is considered an important mechanism of arrhythmia [38, 39], and RyR2 phosphorylation plays a key role in regulation of SR Ca^2+^ release [40–44]. Ryanodine receptor R2 can be phosphorylated by PKA and CaMKII [45–47]. Three phosphorylation sites on RyR2 have been identified: Ser2808, Ser2814, and Ser2030 [46, 48–50]. Although there is no absolute agreement on the specificity of PKA and CaMKII for these phosphorylation sites, it is generally believed that Ser2030 is a PKA target, Ser2814 is a CaMKII target, and Ser2808 can be phosphorylated by PKA or CaMKII [49–53]. Our previous study found that CHSSC can mitigate ischemia-induced increases in the expression of CaMKII and p-CaMKII protein in myocardial tissue [54], which was consistent with the results of our experiments in this study. We also found that the expression of p-RyR2 in myocardial tissue increased after myocardial ischemia in rats, and this increased expression was mitigated by CHSSC. Our results indicated that CHSSC may induce antiarrhythmic effects by regulating the activation of the CaMKII/RyR2/p-RyR2 pathway, resulting in closing of the RyR2 channel, regulation of release of SR Ca^2+^, and reduced intracellular Ca^2+^ levels.

The article "Chai-Hu-San-Shen Capsule Ameliorates Ventricular Arrhythmia Through Inhibition of the CaMKII/FKBP12.6/RyR2/Ca2+ Signaling Pathway in Rats with Myocardial Ischemia" was published in 2022. Journal: Evid Based Complement Alternat Med.

Chronic PKA phosphorylation of RyR2 at Ser2808 results in depletion of Calstabin2 and SR Ca^2+^ leakage, which is one of the earliest described pathological mechanisms of Ca^2+^ leakage that contributes to ventricular arrhythmias [46]. Impairment of the interaction between RyR2 and the 12.6-kDa FK506 binding protein (FKBP12.6) is also an important mechanism of arrhythmia [55, 56]. Studies have shown that PKA phosphorylates RyR2 at Ser2808, which results in dissociation of the RyR2-FKBP12.6 complex, and altered Ca^2+^ channel open probability [46]. In contrast, CaMKII-dependent phosphorylation of RyR2 does not alter FKBP12.6-RyR2 affinity [57]. However, our study showed that after myocardial ischemia, both RyR2 (Ser2814) and RyR2 (Ser2808) were phosphorylated, and the FKBP12.6-RyR2 complex dissociated even when activation of PKA was inhibited. Furthermore, activation of the Ser2808 phosphorylation site on RyR2 after myocardial ischemia was significantly inhibited following treatment with CHSSC, while phosphorylation at Ser2814 was not significantly inhibited, and dissociation of the FKBP12.6-RyR2 complex was inhibited. These results may be related to the activation of CaMKII after myocardial ischemia. Studies have shown that phosphorylation at Ser2808 on RyR2 can occur in response to PKA or CaMKII [49, 51], and the hyperphosphorylation of Ser2808 by CaMKII directly disrupts the binding of FKBP12.6 to RyR2, and can lead to arrhythmias. Furthermore, the expression levels of RyR2 and FKBP12.6 were shown to be decreased in heart failure, while CaMKII expression was increased by 50–100%, and phosphorylation at PKA-specific sites was decreased and phosphorylation at CaMKII-specific sites was increased during this process [58]. Wang et al. have found that the size of the ventricular chamber was enlarged and systolic function was decreased in systolic heart failure. These changes coincided with increased SR Ca^2+^ leakage, and the total amount of FKBP12.6 and FKBP12.6-RyR2 complex increased, and the expression and activity of PKA and CaMKII at their RyR2 phosphorylation sites increased [59]. These results indicated that RyR2 phosphorylation by CaMKII was involved in regulation of dissociation of the FKBP12.6-RyR2 complex. These studies and our data showed that activated CaMKII can regulate the affinity of the FKBP12.6-RyR2 complex through phosphorylation of RyR2 (Ser2814) and/or RyR2 (Ser2808), and CHSSC may reduce phosphorylation of RyR2 (Ser2814) and/or RyR2 (Ser2808) (mainly RyR2 Ser2808) through inhibition of the activation of CaMKII following myocardial ischemia. Treatment with CHSSC may prevent dissociation of the FKBP12.6-RyR2 complex, resulting in reduced intracellular Ca^2+^ content in cardiomyocytes, and protection against arrhythmia.

The article "Chai-Hu-San-Shen Capsule Ameliorates Ventricular Arrhythmia Through Inhibition of the CaMKII/FKBP12.6/RyR2/Ca2+ Signaling Pathway in Rats with Myocardial Ischemia" was published in 2022. Journal: Evid Based Complement Alternat Med.

There were several limitations to our study. First, we did not evaluate PKA, FKBP12.6, or the FKBP12.6-RyR2 complex *in vivo*. Second, as arrhythmia is a complex disease, the isolation of primary myocardial cells from animals may provide additional insights into the pathological processes that occur in arrhythmia. However, isolation of primary cardiomyocytes is very difficult, and H9C2 cells are a generally accepted model for evaluation of cardiomyocyte biochemistry. Since H-89 has been demonstrated to effectively inhibit PKA phosphorylation [60–63], the expression levels of PKA and p-PKA were not evaluated in this study to confirm that PKA activity was inhibited. This study showed that the occurrence of arrhythmia after ischemia was closely related to phosphorylation of RyR2 (Ser2808) and RyR2 (Ser2814) by CaMKII, which promoted dissociation of the FKBP12.6-RyR2 complex, and increased intracellular Ca^2+^ content. However, determination of the specific roles of phosphorylation of RyR2 (Ser2808) and RyR2 (Ser2814) in arrhythmia requires further investigation.

## 5. Conclusion

In conclusion, our results showed that CHSSC induced antiarrhythmic effects by down-regulating the expression of CaMKII and p-CaMKII after myocardial ischemia through inhibition of phosphorylation of p-RyR2 (Ser2808) and p-RyR2 (Ser2814) (mainly through inhibition of RyR2Ser2808 phosphorylation), which resulted in inhibition of dissociation of the FKBP12.6-RyR2 complex, and reduced intracellular Ca^2+^ concentration. We also showed that under the condition of myocardial ischemia, CaMKII is not only involved in regulating the phosphorylation of Ser2808 site on RyR2 but Ser2814 site may be, in addition, Ser2808 site probably the main site of CaMKII acting on RyR2 under this condition.

The article "Chai-Hu-San-Shen Capsule Ameliorates Ventricular Arrhythmia Through Inhibition of the CaMKII/FKBP12.6/RyR2/Ca2+ Signaling Pathway in Rats with Myocardial Ischemia" was published in 2022. Journal: Evid Based Complement Alternat Med.

## Figures and Tables

**Figure 1:** Effect of CHSSC on electrocardiograms in rats with myocardial ischemia. (a) Representative electrocardiogram from the sham operation group. (b) Representative electrocardiogram from the model group. (c) Representative electrocardiogram from the CHSSC treatment group. (d) Representative electrocardiogram from the KN-93 treatment group. *N* = 6 rats per group.

**Figure 2:** Effect of CHSSC on the expression of CaMKII, p-CaMKII, RyR2, and p-RyR2 in rats with myocardial ischemia. (a) Western blot analysis of the expression levels of p-CaMKII, CaMKII, and RyR2. Glyceraldehyde 3-phosphate dehydrogenase was used as the loading control. (b) Quantitative analysis of the relative expression levels of p-CaMKII. (c) Quantitative analysis of the relative expression levels of CaMKII. (d) Quantitative analysis of the relative expression levels of p-RyR2. (e) Quantitative analysis of the relative expression levels of RyR2. *N* = 3 mice per group. All data are expressed as means ± SD. ^*∗*^*P* < 0.05, ^*∗∗*^*P* < 0.01, ^*∗∗∗*^*P* < 0.001 vs. the sham operation group; ^#^*P* < 0.05, ^##^*P* < 0.05, ^###^*P* < 0.001 vs. the model group.

**Figure 3:** Effect of CHSSC on intracellular Ca^2+^ content in ischemic H9C2 cells. (a) Flow cytometry scatter plot from the sham operation group. (b) Flow cytometry scatter plot from the model group. (c) Flow cytometry scatter plot from the CHSSC treatment group. (d) Flow cytometry scatter plot from the KN-93 treatment group. (e) Quantitative analysis of Ca^2+^ content in each group. *N* = 3 samples per group. All data are expressed as means ± SD. ^*∗*^*P* < 0.05, ^*∗∗*^*P* < 0.01, ^*∗∗∗*^*P* < 0.001 vs. the sham operation group; ^#^*P* < 0.05, ^##^*P* < 0.05, ^###^*P* < 0.001 vs. the model group.

**Figure 4:** Effects of CHSSC on the expression of RyR2, p-RyR2 (Ser2808), and p-RyR2 (Ser2814) in ischemic H9C2 cells. (a) Western blot analysis of the expression levels of RyR2, p-RyR2 (Ser2808), and p-RyR2 (Ser2814). Glyceraldehyde 3-phosphate dehydrogenase was used as the loading control. (b) Quantitative analysis of the relative expression levels of RyR2, p-RyR2 (Ser2808), and p-RyR2 (Ser2814) in each group. *N* = 3 samples per group. All data are expressed as means ± SD. ^*∗*^*P* < 0.05, ^*∗∗*^*P* < 0.01, ^*∗∗∗*^*P* < 0.001 vs. the control + H-89 group; ^#^*P* < 0.05, ^##^*P* < 0.05, ^###^*P* < 0.001 vs. the model + H-89 group.

**Figure 5:** Effect of CHSSC on the interaction between FKBP12.6 and RyR2 in ischemic H9C2 cells. (a) Co-immunoprecipitation was used to evaluate the interaction between FKBP12.6 and RyR2. (b) Quantitative analysis of the level of RyR2/FKBP12.6 in each group. *N* = 3 samples per group. All data are expressed as means ± SD. ^*∗*^*P* < 0.05, ^*∗∗*^*P* < 0.01, ^*∗∗∗*^*P* < 0.001 vs. the control + H-89 group; ^#^*P* < 0.05, ^##^*P* < 0.05, ^###^*P* < 0.001 vs. the model + H-89 group.

The article "Chai-Hu-San-Shen Capsule Ameliorates Ventricular Arrhythmia Through Inhibition of the CaMKII/FKBP12.6/RyR2/Ca2+ Signaling Pathway in Rats with Myocardial Ischemia" was published in 2022. Journal: Evid Based Complement Alternat Med.

**Table 1:** Chinese herbs of CHSSC.

Chinese name	English name	Latin name	Drug proportion
Gan Cao	GLYCYRRHIZA RADIX ET RHIZOMA	Glycyrrhiza uralensis Fisch.	6
Huang Qin	SCUTELLARIAE RADIX	*Scutellaria baicalensis Georg*i	6
Dan Shen	SALVIAE MILTIORRHIZAE RADIX ETRHIZOMA	*Salvia miltiorrhiza* Bge.	10
Fa Ban Xia	PINELLIAE RHIZOMA PREPARATUM	*Pinellia ternata* (Thun.)	10
Ku Shen	SOPHORAE FLAVESCENTIS RADIX	Sophora flavescens Ait.	10
Qing Hao	ARTEMISIAE ANNUAE HERBA	*Artemisia annua L*.	10
Dang Shen	CODONOPSIS RADIX	*Codonopsis pilosula* (Franch.) Nannf.、	15
Chai Hu	BUPLEURI RADIX	*Bupleurum chinense* DC.	15

**Table 2:** Results of electrocardiogram in each group.

Groups	n	VPB		VT		VF	
		Frequency (times)	First occurrence time (min)	Frequency (times)	Duration time (min)	Frequency (times)	Duration time (min)
Sham	6	0	0	0	0	0	0
Model	6	17.7 ± 1.3	4.4 ± 0.4	14.0 ± 1.0	15.2 ± 0.4	6.7 ± 0.7	4.8 ± 1.0
CHSSC	6	9.7 ± 0.9^*∗∗∗*^	6.6 ± 0.5^*∗∗∗*^	7.0 ± 3.8^*∗*^	9.4 ± 5.0^*∗∗∗*^	0	0
KN-93	6	7.6 ± 0.5^*∗∗∗*^	7.1 ± 0.8^*∗∗*^	4.0 ± 2.3^*∗∗∗*^	6.4 ± 3.5^*∗∗∗*^	0	0

**Table 3:** The mean OD value and survival rate of H9C2 cell in each group.

Groups	Normal group	5% medicated plasma group	10% medicated plasma group	20% medicated plasma group	5% nonmedicated plasma group	10% nonmedicated plasma group	20% nonmedicated plasma group
Mean OD value	1.2534	1.2531	1.0823	0.3215	1.2671	1.2568	1.1287
Survival rate	100.00%	99.98%	86.35%	25.55%	101.09%	100.27%	90.05%

## Data Availability

The data sets used and analyzed for this article will be made available from the authors upon reasonable request.

## Abbreviations

CHSSC: Chai-hu-san-shen capsule
TCM: Traditional Chinese medicine
SR: Sarcoplasmic reticulum
ER: Endoplasmic reticulum
RyRs: Reynolds ryanodine receptors
PKA: Protein kinase A
FKBP: FK506 binding protein
CaM: CalModulin
CaMKII: Calmodulin-dependent protein kinase II
VPB: Ventricular premature beat
VT: Ventricular tachycardia
VF: Ventricular fibrillation.
